# Clinical Usage of Different Doses of Cis-Atracurium in Intracranial Aneurysm Surgery and Its Effect on Motor-Evoked Potentials

**DOI:** 10.1155/2022/5910019

**Published:** 2022-06-28

**Authors:** Zhongyuan Qiao, Rong Fan

**Affiliations:** Anesthesiology Department, The First Affiliated Hospital of Northwest University (Xi'an No. 1 Hospital), Xi'an, 710000 Shaanxi, China

## Abstract

The objective of this work was to investigate the effect of different doses of cis-atracurium on patients undergoing general anesthesia induction (GAI) during intracranial aneurysm surgery (ICAS). In this work, 90 patients who underwent ICAS under the elective motor-evoked potential (MEP) monitoring in the First Affiliated Hospital of Northwest University (Xi'an No. 1 Hospital) from January 2021 to May 2022 were enrolled as the research objects. Randomly, they were rolled into a S1 group (30 cases, 2 times 95% effective dose (ED95) cis-atracurium), a S2 group (30 cases, 3 times ED95 cis-atracurium), and a S3 group (30 cases, 4 times ED95 cis-atracurium). The endotracheal intubation conditions, the train-of-four (TOF) rate (TOFR), body movement, and spontaneous breathing were compared among the three groups of patients. The results showed that the MEP inhibition time of the patients in the S3 group was much longer than that of the S1 and S2 groups, but it showed no significant difference between the S1 group and S2 group (*P* > 0.05). The good rates of endotracheal intubation conditions in the S2 group (100%) and S3 group (100%) were obviously higher than the rate in the S1 group (43.33%). The TOFRs of patients in S2 and S3 groups at time t2 and t3 were lower obviously to that at time t0, while the TOFRs of patients in S3 group at time t2 and t3 were still lower in contrast to the S2 group (*P* < 0.05). The mean arterial pressure (MAP) and heart rate (HR) of patients in all groups were lower at t1, t2, and t3 than at t0 (*P* < 0.05), while the differences among different groups were not remarkable (*P* > 0.05). Finally, using 3 times ED95 cis-atracurium for GAI could reduce the risk of intraoperative body movement and spontaneous breathing, as well as the residual degree of muscle relaxation, in patients with ICAS, without affecting MEP monitoring, improving endotracheal intubation conditions, and increasing safety during open neurosurgery operations.

## 1. Introduction

Intracranial aneurysm generally refers to the abnormal bulge of the intracranial artery wall, which is the first cause of subarachnoid haemorrhage [1]. Due to the weak structure and poor elasticity of the blood vessel wall of a cerebral aneurysm, it is possible that the rupture of the cerebral aneurysm may occur when the mean arterial pressure (MAP) increases during emotional agitation, forced defecation, fatigue, etc., so the incidence rate is extremely high. Outside of the cerebral blood arteries, the incidence of cerebral haemorrhage (subarachnoid haemorrhage) produced by cerebral aneurysm is currently second only to cerebral thrombosis and hypertensive cerebral haemorrhage, and the fatality rate is first [2–4]. Most intracranial aneurysms occur in middle-aged and elderly women between the ages of 40 and 60. At present, the etiology of intracranial aneurysms is still unclear. Most scholars believe that intracranial aneurysms are caused by local congenital defects in the intracranial arterial wall and increased intraluminal pressure. Hypertension, cerebral arteriosclerosis, and vasculitis are associated with the occurrence and development of aneurysms [5, 6]. Intracranial aneurysms are usually minor and cause no symptoms. Aneurysms are discovered in two ways: when they rupture and bleed, creating a severe headache or coma, and when they compress and create a sequence of symptoms [7]. Although the process of aneurysm rupture and bleeding lasts only a few seconds, it can bring a series of serious consequences, so once the intracranial aneurysm lesion is detected, it should be treated as soon as possible [8].

Clinical treatment of intracranial aneurysms mainly includes open surgical treatment (clamping, wrapping), endovascular interventional treatment (coils, blood flow guide devices, liquid embolic agents, stents, etc.), and conservative treatment to control the risk factors [9, 10]. Clipping is to select the appropriate aneurysm to clip the aneurysm according to the orientation of the aneurysm and the length of the aneurysm neck. It is a common method for the treatment of intracranial aneurysms. If it is closed, aneurysm wrapping will be used. Endovascular interventional therapy is a new alternative treatment for inoperable patients, mainly by implanting coils, stents, balloons, liquid glue, and other materials for aneurysm treatment [11–13]. Interventional therapy, on the other hand, has a dismal prognosis. Some people, for example, will have increased blood viscosity. When the blood arteries in the head narrow and spasm, the blood flow rate slows, increasing the risk of a head blood vessel infarction. In addition, patients may also experience hemiplegia, aphasia, intellectual disability, and movement disorders [14–16]. Unfortunately, these conventional treatments all have many difficulties for giant intracranial aneurysms, such as huge aneurysm, thin wall, easy rupture and bleeding, wide aneurysm neck, difficult or impossible to clip. It is not suitable for tamponade, or the pituitary gland is still compressed after tamponade, and it is difficult to improve the symptoms of patients [17, 18].

The motor-evoked potential (MEP), which can reflect the integrity of the descending pathway of anterior spinal cord motor conduction and is used clinically to assess the integrity of the patient's motor function in real time, is one of the key elements to be monitored in neurosurgery. As a result, improving the accuracy of MEP intraoperative monitoring is an area that requires focus [19, 20]. There are many factors that affect MEP, such as anesthesia drugs, pacemakers, and surgical operations, among which anesthesia drugs have the greatest impact. Cis-atracurium is a synthetic bisquaternary ammonium ester type benzyl isoquinoline compound, which is a medium-acting nondepolarizing muscle relaxant, can act through competitive binding with cholinergic receptors, has a rapid onset of action, and has a good muscle relaxation effect, and is widely used in clinical anesthesia [21–23]. As a result, 90 ICAS patients who underwent MEP monitoring in our hospital were chosen as research subjects and divided into three groups: S1 (2 times the 95 percent effective dose (ED95) cis-atracurium), S2 (3 times ED95 cis-atracurium), and S3 (4 times ED95 cis-atracurium), each having 30 cases [24, 25]. It compared the general data, endotracheal intubation conditions, hemodynamic indexes, respiratory function indexes, train-of-four (TOF) ratio (TOFR), body movement, and spontaneous breathing conditions of the three groups of patients, so as to deeply analyze the effects of different doses of cis-atracurium on GAI of patients with ICAS.

## 2. Materials and Methods

### 2.1. Research Objects

90 ICAS patients who underwent MEP monitoring in the First Affiliated Hospital of Northwest University (Xi'an No. 1 Hospital) from January 2021 to May 2022 were selected as the research subjects. The experiment had been approved by the Ethics Committee of the First Affiliated Hospital of Northwest University (Xi'an No. 1 Hospital), and the informed consents had been obtained from all patients and their families

Patients enrolled had to meet the following criteria: patients who were older than 18 years old, patients who were determined as American Society of Anesthesiologists (ASA) grade I or II, persons with normal body temperature, patients with complete clinical data, and patients with normal communication.

Patients satisfying below conditions had to be excluded from this work: patients with moderate to severe anemia; patients with difficult airway; patients with infection at the monitoring site; patients with severe heart, liver, and kidney disease; patients complicated with mental illness; patients who are allergic to anesthetics; and patients with malignant tumors or other malignant diseases.

### 2.2. Grouping of Objects

The patients were divided into 30 cases in the S1 group, 30 cases in the S2 group, and 30 cases in the S3 group by a random number table method. Patients in group S1 were treated with 2 times the 95% effective dose (ED95) cis-atracurium; patients in group S2 were treated with 3 times ED95 cis-atracurium; and patients in group S3 were treated with 4 times ED95 cis-atracurium.

### 2.3. Anesthesia Method

Firstly, before the surgery, the patient was allowed to fast for 8 hours and water for 5 hours. The electrocardiogram, heart rate (HR), MAP, and other physical indicators of patients should be monitored after they entered the operation room. They all received intravenous anesthesia, intravenous infusion of 0.4 mg of scopolamine before anesthesia. Secondly, during the anesthesia, 0.04 mg/kg of midazolam and 1.5 mg/kg of propofol were intravenously injected in sequence. After the patient lost consciousness, 0.4 *μ*g/kg of sufentanil was intravenously injected, and electrophysiological monitor was performed. Thirdly, different doses of cis-atracurium were intravenously injected to the corresponding patients, and the tracheal intubation was performed through the mouth (dyclonine hydrochloride mucilage was applied to the surface of the tracheal tube) after the drug took effect. Fourthly, it could select the appropriate size catheter according to the individual situation of the patient, adjust the depth of tracheal intubation by auscultation, and perform mechanically controlled ventilation after fixation. Respiratory parameters were set as follows: the tidal volume was 8.5-10.5 mL/kg, the respiratory rate was 10-12 times/min, and the oxygen flow was 1.5 L/min. Fifthly, during the surgery, the end-tidal carbon dioxide should be maintained at a level of about 35 mmHg, and the fluid infusion rate should be adjusted according to the patient's MAP and HR in real time to maintain hemodynamic balance. Half an hour before the end of surgery, the patient should be given 4 mg of dezocine and 0.02 mg/kg of tropisetron. Propofol and sufentanil injections were stopped 10 minutes before the end of surgery. After the patient regained spontaneous breathing, neostigmine and atropine were administered intravenously, and tracheal extubation was performed after the patient was completely awake.

### 2.4. MEP Monitoring

MEP monitoring was performed using a 32-channel bioelectrophysiological signal analysis system XLTEK32 (GE, USA). Firstly, the abductor pollicis brevis muscle, the abductor pollicis muscle of the upper extremity, and the abductor pollicis muscle of the lower extremity were selected as the monitoring sites, and the spiral electrode was used as the scalp stimulation electrode. The line was placed on the shoulders of the changer. The stimulation parameters were set as follows: the stimulation intensity was about 120 V, the stimulation frequency was 5-10 times, the stimulation interval was 2-3.5 ms, and the pulse was 45 *μ*s. It should record the compound muscle action potential at the corresponding muscle position at the speed of 8 ms/div, the filter of 50-2500 HZ, and the display gain of 45 *μ*v/div. The electrodes can be stimulated after the intravenous injection of cis-atracurium.

### 2.5. Intraoperative Emergency Response Measures

The following are the emergency response measures: (1) If the patient recovered spontaneous breathing during the operation, the ventilator can be adjusted to manual assisted ventilation mode, and about 30 mg of propofol can be intravenously infused. It can adjust to the mechanically controlled ventilation mode when the patient has no spontaneous breathing. (2) If the patient had body movement during the surgery, it could inject about 30 mg of propofol and temporarily stop the MEP monitoring. (3) When the patient's MAP decreased by more than 30% (compared to the baseline value), appropriate fluid replacement was required, and norepinephrine bitartrate (3 *μ*g single injection) was used as appropriate; if the patient's MAP increased by more than 30% (compared to the baseline value), which can deepen the degree of anesthesia and use vasoactive drugs as appropriate. (4) If the patient's HR decreased by more than 30% (compared to the basal value), it could give the patient 0.4 mg of atropine; if the patient's HR increased by more than 30% (compared to the basal value), appropriate fluids can be added to maintain a sufficient degree of anesthesia and as appropriately adopt the *β*-blockers.

### 2.6. Observation Indexes

The general information of the patients (age, gender, height, weight, hypertension, diabetes, and coronary heart disease (CHD)) was collected. MAP, HR, pulse oxygen saturation (SpO_2_), partial pressure of carbon dioxide in end-expiratory gas (PETCO_2_), and peak airway pressure (Peak) were recorded at different times (when entering the room (t0), immediately after endotracheal intubation (t1), 5 minutes after endotracheal intubation (t2), and release of MEP waveform (t3)). The TOF-Watch SX acceleration muscle relaxation monitor was used to evaluate the residual effect of the patient's muscle relaxation, and TOFR was calculated. Cooper's scoring method [22] was adopted to evaluate endotracheal intubation conditions, including the sum of three scores: laryngoscopy, glottis opening, and closing and intubation response. The suppression time and operation time of the patient's MEP waveform were recorded.

### 2.7. Statistical Methods

SPSS19.0 was used for data processing in this work. Measurement data were expressed in the form of mean ± standard deviation ($\bar{x}\pm s$), and enumeration data were expressed as percentage (%). Pairwise comparisons were made using one-way ANOVA. The difference was statistically significant at *P* < 0.05.

## 3. Results and Discussion

### 3.1. Comparison on General Data of Patients in Different Groups

As shown in Figure 1 below, there were no statistically obvious differences in the ratio of males and females, average age, body mass index (BMI), hypertension, diabetes, and CHD among three groups (*P* > 0.05).

### 3.2. Comparison of Perioperative Conditions of Patients

As shown in Figure 2 below, the operation time showed no great difference among the S1, S2, and S3 groups (*P* > 0.05). The MEP inhibition time of the S3 group was the longest among all groups (*P* < 0.05), while it showed no obvious different between the S1 and S2 groups (*P* > 0.05).

As illustrated in Figure 3, the pairwise comparison of MAP and HR at t0 in the three groups of patients showed the difference was not statistically notable (*P* > 0.05); those at t1, t2, and t3 were lower than at t0 time (*P* < 0.05); and no remarkable difference was found among the three groups at t1, t2, and t3 (*P* > 0.05).

As demonstrated in Figure 4, the pairwise comparisons of SpO_2_, PETCO_2_, and peak among all groups showed no obvious difference at all time points (*P* > 0.05).

As given in Figure 5, the TOFRs of the three groups of patients at time t0 were not different greatly (*P* > 0.05); the TOFRs in the S2 groups and the S3 group at time t2 and t3 decreased than those before surgery (*P* < 0.05), while those in the S3 group were lower in contrast to those in the S2 group at both t2 and t3 (*P* < 0.05).

As shown in Tables 1 and 2, patients in group S1 did not experience body movement or spontaneous breathing at time t0, t1, and t2, while at t3, 3 patients had body movement and 2 patients had spontaneous breathing. Patients in groups S2 and S3 did not experience body movement or spontaneous breathing at all time points.

Figure 6 shows the comparison of the dosage of propofol and sufentanil among the three groups of patients. The dosage of propofol in patients with S1 was 734.65 ± 102.34 mg, and the dosage of sufentanil was 2.04 ± 0.25 mg. The dosages of propofol and sufentanil in the S2 group were 679.25 ± 97.54 mg and 1.87 ± 0.18 mg, respectively; the dosages of propofol and sufentanil in S3 group were 678.05 ± 99.25 mg and 1.79 ± 0.38 mg, respectively. The analysis showed no visible difference in the doses of propofol and sufentanil among the three groups of patients (*P* > 0.05).

### 3.3. Comparison of Intraoperative Endotracheal Intubation Conditions

Figure 7 shows the comparison of the endotracheal intubation conditions of the three groups of patients. It showed that the patients in the S1 group had excellent endotracheal intubation circumstances in six cases, good in seven, moderate in eleven, and poor in six. The endotracheal intubation conditions of the patients in the S2 group were excellent in 23 cases, good in 7 cases, moderate in 0 cases, and poor in 0 cases. In the S3 group, the endotracheal intubation conditions were excellent in 24 cases, good in 6 cases, moderate in 0 cases, and poor in 0 cases. The analysis showed that the excellent and good rates of endotracheal intubation conditions of patients in S2 group (100%) and S3 group (100%) were absolutely higher in contrast to those in S1 group (43.33%), showing statistically visible differences (*P* < 0.05).

## 4. Discussion

Intracranial aneurysm is a clinical disease with a very high morbidity and mortality rate. Although aneurysm is not a tumor, it is much more dangerous than a tumor [23, 24]. However, because the human brain is such a complicated organ, even minor injury might impair the patient's neurological function, so the procedure must be done with extraordinary precision. In ICAS, neurophysiological monitoring is the gold standard for detecting nerve injury induced by various variables in time for scientific intervention [25, 26]. Muscle relaxants are a major factor affecting the accuracy of MEP monitoring. Therefore, this work included 90 ICAS patients who underwent MEP monitoring in our hospital from January 2021 to May 2022 and divided the patients into a S1 group (2 times ED95 cis-atracurium), a S2 group (3 times ED95 cis-atracurium), and a S3 group (4 times ED95 cis-atracurium) for comparative analysis, with 30 cases in each group. Firstly, the basic data of the three groups of patients were compared, and it was found that the ratio of males and females, average age, BMI, hypertension, diabetes, and CHD in the S1, S2, and S3 groups were not greatly different (*P* > 0.05). This provides a reliable basis for follow-up research.

Then, it analyzed the perioperative conditions of the three groups of patients. Firstly, difference in the operation time between the three groups of patients in the S1, S2, and S3 groups was not great (*P* > 0.05). This is similar to the findings of Pressman et al. [27], indicating that the dose of cis-atracurium dies not differ in terms of ICAS length. The MEP inhibition time of the S3 group was the longest to the S1 and S2 groups; it was not greatly different between the S1 and S2 groups (*P* > 0.05). This suggests that when the induction dose is increased from 2 times ED95 cis-atracurium to 3 times ED95 cis-atracurium, the inhibition time of MEP waveform will not be significantly prolonged; and the 4 times ED95 cis-atracurium could result in a substantial prolongation of the suppression time of the MEP waveform. Such results suggest that the doses of 2 times ED95 cis-atracurium and 3 times ED95 cis-atracurium will not affect MEP and are suitable for use in neurosurgery ICAS. The comparison on endotracheal intubation conditions of the three groups of patients revealed that in the S1 group it was excellent in 6 cases, good in 7 cases, moderate in 11 cases, and poor in 6 cases; it was excellent in 23 cases, good in 7 cases, fair in 0 cases, and poor in 0 cases in S2 group; and it was excellent in 24 cases, good in 6 cases, moderate in 0 cases, and poor in 0 cases in S3 group. The analysis showed that the excellent and good rates of endotracheal intubation conditions in the S2 group and the S3 group (both were 100%) were absolutely higher compared with the S1 group (43.33%), and the differences were statistically notable (*P* < 0.05). Such results suggest that 2 times ED95 cis-atracurium doses had poor endotracheal intubation conditions. Furthermore, at time t0, t1, and t2, patients in the S1 group did not have any body movement or spontaneous breathing. Three patients experienced body movement, and two had spontaneous breathing at time t3. At t0, t1, t2, and t3, no body movement or spontaneous breathing occurred in groups S2 and S3. Such results further indicate that 3 times ED95 cis-atracurium and 4 times ED95 cis-atracurium are better than 2 times ED95 cis-atracurium for maintaining the patient's intraoperative condition [28]. Based on the above results, it can be known that the anesthetic dose of 3 times ED95 cis-atracurium is the most suitable for ICAS.

During the surgery, the reduction of MAP in patients often exceeds the clinical standard and affects the hemodynamics of patients, so intraoperative monitoring of hypotension is very important [29]. It was found in this work that the MAP and HR of the three groups of patients at t1, t2, and t3 were decreased compared with those at t0, while the differences between groups at t1, t2, and t3 were not statistically obvious (*P* > 0.05). The use of intraoperative anesthetics can make the MAP of the patients drop to a certain extent, which is a normal clinical manifestation. The results indicate that the dose of cis-atracurium does not affect the hemodynamic changes of the patients. In addition, this work found that the SpO_2_, PETCO_2_, and peak at t1, t2, and t3 of the three groups of patients were not observably different from those at t0 (*P* > 0.05). No statistically remarkable difference among the three groups in SpO_2_, PETCO_2_, and peak was found at time t1, t2, and t3 (*P* > 0.05). SpO_2_, PETCO_2_, and peak are all main indicators of respiratory function monitoring during surgery. PETCO_2_ refers to the carbon dioxide partial pressure or carbon dioxide concentration in the mixed alveolar air exhaled at the end of expiration. It is often used to evaluate patients' ventilatory function, circulatory function, pulmonary blood flow, alveolar ventilation, subtle repeated inhalation, and the patency of the entire airway and breathing circuit. SpO_2_ is the percentage of oxyhemoglobin in the blood to the total hemoglobin volume, which is used to assess the patient's breathing and circulation. Peak airway pressure is the highest pressure experienced during ventilator insufflation, and it is determined by lung compliance, airway resistance, tidal volume, and other factors [30]. As a result, the findings suggest that the incidence of intraoperative respiratory depression in patients is unrelated to the use of various cis-atracurium doses and that the analysis could be induced by intravenous injections of propofol and sufentanil. The TOFRs of patients in the S2 and S3 groups at time t2 and t3 were much lower than those at time t0, while the TOFRs of patients in group S3 at time t2 and t3 were not as high as those in group S2, and the differences were obvious (*P* < 0.05). Such conclusions are similar to the results of Ding et al. [31]. The TOFR represents the degree of blockade of the presynaptic receptors, indicating that 2 times ED95 cis-atracurium and 3 times ED95 cis-atracurium can reduce the residual degree of muscle relaxation and improve intracranial surgical openness without affecting MEP monitoring, improving the safety during the ICAS.

## 5. Conclusions

From January 2021 to May 2022, 90 ICAS patients underwent MEP monitoring at Northwest University's First Affiliated Hospital (Xi'an No. 1 Hospital). The patients were randomly assigned to one of three groups: S1 (2 times ED95 cis-atracurium), S2 (3 times ED95 cis-atracurium), and S3 (4 times ED95 cis-atracurium). The general data, endotracheal intubation conditions, TOFR, body movement, spontaneous breathing, and hemodynamic indicators were compared among the three groups of patients. Finally, it was found that GAI using 3 times ED95 cis-atracurium can reduce the risk of intraoperative body movement and spontaneous breathing and the residual degree of muscle relaxation in patients with intracranial aneurysm and improve endotracheal intubation conditions without affecting MEP monitoring and hemodynamics, enhancing the safety during open neurosurgery procedures. However, the sample size of patients included was small, and the source was single, which may have some influence on the results. Moreover, no follow-up observation of patients' postoperative conditions was conducted, and there was a lack of patient prognosis data using different doses of cis-atracurium. As a result, in future studies, it will consider using more case data in the analysis to further investigate the best cis-atracurium dose. In conclusion, the results of this work could provide a reference for the dose selection of GAI muscle relaxants in ICAS.

## Figures and Tables

**Figure 1:** Comparison on the general data of patients ((a) is the comparison on number of male and female cases; (b) shows the comparison of the average age and BMI; (c) illustrates the comparison of the ASA classification; (d–f) compare the number of hypertension, diabetes, and CHD, respectively).

**Figure 2:** Comparison of operation time and MEP inhibition time ((a) compares the operation time; (b) compares the MEP inhibition time).

**Figure 3:** Comparison of MAP and HR at different times ((a) compares the MAP, and (b) compares the HR) Note: ∗ indicates *P* < 0.05 compared with the values at time t0.

**Figure 4:** Comparison on SpO_2_, PETCO_2_, and peak ((a–c) compare the SpO_2_, PETCO_2_, and peak, respectively).

**Figure 5:** Comparison of TOF values of three groups of patients at different times. Note: ∗ and ^#^ mean *P* < 0.05 in contrast to the values at t0 and S3 group, respectively.

**Figure 6:** Comparison of the dosage of propofol and sufentanil ((a) shows the comparison of propofol; and (b) illustrates the comparison of sufentanil).

**Figure 7:** Comparison of intraoperative endotracheal intubation conditions among three groups of patients ((a) shows the number of excellent, moderate, and poor cases; (b) shows the excellent and good rate) Note: ∗ indicates that the difference was statistically great compared with the S1 group (*P* < 0.05).

**Table 1:** Statistics on body movement of patients.

Time	S1 group	S2 group	S3 group
t0	30	30	30
t1	0	0	0
t2	0	0	0
t3	3	0	0

**Table 2:** Statistics on spontaneous breathing of patients.

Time	S1 group	S2 group	S3 group
t0	30	30	30
t1	0	0	0
t2	0	0	0
t3	2	0	0

## Data Availability

The data used to support the findings of this study are available from the corresponding author upon request.
